# Factors Influencing the Teaching Intention of Business College Teachers to Fulfill Digital Entrepreneurship Courses

**DOI:** 10.3389/fpsyg.2022.860808

**Published:** 2022-05-03

**Authors:** Tai-Kuei Yu, Cheng-Min Chao, YiJie Wang

**Affiliations:** ^1^Department of Business Administration, National Quemoy University, Kinmen, Taiwan; ^2^Department of Business Administration, National Taichung University of Science and Technology, Taichung, Taiwan; ^3^Faculty of Sociology, Lomonosov Moscow State University, Moscow, Russia

**Keywords:** digital entrepreneurship education, task-technology fit, self-determination theory, positive attitude emotions, partial least square

## Abstract

With the increasing promotion of entrepreneurship in Taiwan’s universities and the establishment of departments of innovation or entrepreneurship management, it has become an emerging trend to encourage college students to become entrepreneurs or participate in entrepreneurial competitions during their undergraduate years. The Internet has stimulated the development and widespread application of new business models and has created a large number of entrepreneurial opportunities. Universities engaged in digital entrepreneurship education over the past have hardly designed a curriculum to teach the content of digital entrepreneurship. This study integrated “task-technology fit,” “self-determination theory,” and “interactive participation,” into its investigation on the teaching intention of business college teachers to develop digital entrepreneurship courses. The sample size was 126 participants. Using partial least squares analysis, the research model represented high internal consistency and confirmed the good reliability of the scales. This study presented that three dimensions of the concept (teachers’ positive attitude emotions, task-technology fit, interactive participation) were highly prioritized in their intention to teach digital entrepreneurship courses. The coefficient of the endogenous variables was 0.503 for positive attitude emotions, 0.571 for task-technology fit, and 0.392 for teaching intention. Based on a quantitative survey on the teaching intention of business college teachers to fulfill digital entrepreneurship courses, this study demonstrated the implications of digital entrepreneurship education issues that are relevant to the role of teacher’s dimension from different viewpoints, and discussed the implications of teaching digital entrepreneurship courses for digital entrepreneurship practices and entrepreneurship education.

## Introduction

There is a very close relationship between innovation and entrepreneurship. Innovation-oriented entrepreneurial activities can provide assistance to economic growth, becoming an important source of competitive advantage, an important way to create wealth and value, and an important force to promote economic and social development (Kakouris and Liargovas, 2021; Ratten and Jones, 2021). Entrepreneurship education, which links together business theory and practice, has become one of the most popular subjects in management education. Kakouris and Liargovas (2021) define entrepreneurship education as a series of education and training activities that try to develop the intention of entrepreneurial behavior, implement entrepreneurship among participants, and promote some factors of entrepreneurial intention. The access to online platforms is now much easier to get than it was a few years ago. Information communication technology (ICT) has created more opportunities for more potential contributors to collaboratively develop new products and service solutions, changing the business competition environment and creating new business strategies, models, and processes (Elia et al., 2020). As for learning activities in the context of digital entrepreneurship education (DEE), scholars (Giones and Brem, 2017; Nambisan, 2017; Kraus et al., 2018; Secundo et al., 2021) have generally believed that learning about digital entrepreneurship involves knowledge acquisition, knowledge structure, skills, and attitudes. These learning activities try to make participants use ICT tools and technologies, take advantage of the low entrepreneurial costs and the large number of potential customers of digital entrepreneurship, thereby discovering entrepreneurial opportunities and executing digital or non-digital entrepreneurial activities. Therefore, DEE relies more on the use of digital technologies in reconfiguring the design and delivery of the learning process in entrepreneurship education. The purpose of its curriculum design is to strengthen the power of education system to integrate the use of digital tools and business capabilities (Rippa and Secundo, 2019; Zaheer et al., 2019; Ratten and Jones, 2021).

The outbreak of COVID-19 has posed a major challenge to entrepreneurship education. The use of digital technologies has increased significantly in virtual and real environments on the Internet, and virtual teamwork is commonly used to promote the accelerated application of digital technologies. As our society has gradually adapted to the needs of digital market transactions, more and more digital innovations and digital service business activities are taking place. However, research in DEE still remains at the early stage of development. It is necessary to teach digital creativity and value innovation in the digital business environment, in order to obtain access to better online businesses. Knowledge related to risks of online business activities plays a key role (Nambisan, 2017; Steininger, 2019; Vorbach et al., 2019; Secundo et al., 2021). DEE enables students to learn the abilities needed to discover new business opportunities in the digitalized generation. For example, entrepreneurial knowledge, the accessibility of entrepreneurial activities, the feasibility of these activities to combine with digital technology, and other entrepreneurship-related abilities are easily acquired through formal education, because they can be developed through teaching and training (Morris et al., 2013; Shabbir et al., 2016; Nambisan, 2017; Vorbach et al., 2019; Kakouris and Liargovas, 2021). Much emphasis should be put on what business literacy teachers need to improve the quality and effectiveness of DEE teaching programs, such as providing individuals with the ability to identify business opportunities and the insight to respond to these opportunities, together with self-esteem, knowledge, processing skills, and entrepreneurs’ spirit. All of these areas take competence development as the major element for development, training, and education (Oosterbeek et al., 2010; Otache, 2019). In knowledge-intensive industries that require knowledge about innovation, digital transformation has led to constant changes in the competitive environment. Therefore, more digital skills combined with entrepreneurial activities can help people develop the creative thinking and the resilience required by the environment digital economy (Jones et al., 2018; Kraus et al., 2018; Ngoasong, 2018; Ratten and Jones, 2021). Indeed, entrepreneurial thinking ability has been taught and trained through education, and qualified individuals have been trained from the perspective of education. By integrating the use of information and communication technology (ICT) into the teaching content of DEE, the skills of digital entrepreneurship can be developed (Karatas and Ozcan, 2010; Guthrie, 2014; Turkdogan, 2019).

Schools can be a place to develop the teaching and learning of creativity. In addition to having entrepreneurial thinking and teaching abilities, teachers must play the role of promoters of entrepreneurship as well as innovators of creativity. As an on-site instructor, teachers will indeed be the key agents to complete this task together with students. Their self-motivation is effective in improving entrepreneurship teaching; it can encourage students to become entrepreneurs (Seikkula-Leino et al., 2010; Fellnhofer, 2019; Ayyildiz and Yilmaz, 2021; Garcez et al., 2021). Teachers participating in DEE should receive long-term and specific training and should have sufficient resources (in terms of money and time) to plan, implement, and evaluate DEE. This will make them aware of their responsibilities, motivate them, and help them understand that the role of teachers has become more important than ever in DEE (Ismail et al., 2018; Iwu et al., 2019; Keyhani and Kim, 2020). The integration of technology with education to innovate teaching practice is regarded as a complex and multi-dimensional process of innovation, which puts forward requirements for teachers’ innovation and professional learning ability (Ismail et al., 2018; Kraus et al., 2018). Teachers may have professional skills and business experiences, but they still need more entrepreneurial practices. Against this background where the technology for teaching and learning has been changing rapidly, Guthrie (2014) discussed the importance of cooperation in teaching between teachers and industry professionals, emphasizing that teachers should actively participate in professional knowledge and curriculum planning. He also stressed that it is necessary for teachers to explain to students all the entrepreneurial concepts as early as possible, in order to show students how entrepreneurial activities may proceed. When students make mistakes upon entering an experiential learning activity, teachers can immediately take corrective measures, give them feedback, and motivate their students.

The establishment, survival, and development of an enterprise are particularly relevant. Knowledge, skills and experience can be learned and improved through education (Kakouris and Liargovas, 2021; Ratten and Jones, 2021), and the components of entrepreneurial competence can be taught through business activities. There are four categories of competences most consistently identified in literature review: entrepreneurship competences, business and management competences, human relations competences, and interpersonal competences (Mitchelmore and Rowley, 2010; Bamiatzi et al., 2015). The universal use of digital technology has also been promoted in entrepreneurship education. Through the use of different virtual platforms, the reuse of digital content and the integration of new complementary technologies bring forth new technologies that have has become a unique, innovative service for its business models and operations. The digital transformation of goods and services has affected the teaching and learning methods of entrepreneurship (Grégoire and Shepherd, 2012; Ngoasong, 2018; Garcez et al., 2021). Transforming business ideas into successful start-ups requires a collection of interdisciplinary information as well as sufficient business and management literacy. Through specialized digital entrepreneurship modules, digital transformation, and the development of entrepreneurial skills, students are able to focus on identifying and pursuing digital opportunities as well as acquiring a range of business and entrepreneurial knowledge and skills (Al-Atabi and DeBoer, 2014; Geissinger et al., 2019; Vinogradova et al., 2019; Ratten and Jones, 2021; Secundo et al., 2021).

The three basic motivations of digital entrepreneurship are revitalization, integration, and value creation. To adapt to the social needs of continuous digital transformation, companies that have become slow in their business paces need to use ICT tools to rejuvenate their operations. Modifying ICT can provide companies with a way to change their *status quo* and place more emphasis on innovation, which means a new way to integrate and adjust existing operations, thereby generating key value creation for corporate activities. Despite the differences in business focus, it is useful to integrate value creation into all business decisions (Giones and Brem, 2017; Guthrie, 2014). Teachers’ willingness to change their teaching and learning is closely related to the following elements: their personal reflections on the adoption and promotion of new technologies; the professional development of technology on the part of teachers, their colleagues, or experts inside and outside their institutions; and their acceptance and adoption of new technology (Oosterbeek et al., 2010; Guthrie, 2014; Kraus et al., 2018; Nambisan, 2017). pointed out that teaching in new professional fields may force teachers and educators to reflect on their beliefs in teaching and learning, which is essential for their adaptation to true teaching activities integrated with ICT; yet, they are also actively seeking new technical support and cooperation to maintain these changes. As the impact of digital transformation has become widely present in most industries and different types of companies, digital technology has become a promoter of entrepreneurial activities (Nambisan, 2017; von Briel et al., 2018; Steininger, 2019; Zaheer et al., 2019; Elia et al., 2020; Sahut et al., 2021). In addition to digital entrepreneurship embedded with the importance of educational practice, this study explored how to promote the teaching intention of business college teachers to fulfill digital entrepreneurial activities from the perspectives of teachers’ demand for self-professional growth and new business opportunities brought by digital technology and the Internet. The remaining of this study is organized as follows. Section “Literature review” discusses its research model and research hypotheses based on the empirical cases of Self-determination theory and Task Technology fit, while section “Data and Methods” describes its research methods related to research procedures and data analysis; section “Results” outlines its data analysis techniques and describes statistical results; section “Discussion” reviews the differences between empirical results and past research, states some theoretical and managerial implications, and describes the limitations associated with this study; finally, section “Conclusions” brings forth the important implications of this study.

## Literature Review

### Self-Determination Theory

Self-determination theory (SDT) provides a conceptual framework for the study of individual behavior motivation, describes individual autonomy and control over the behavior, and identifies the driven factors of individual behavior. It has been proven that individual behavioral and behavior intention will be affected by motivation and will affect whether personal behavior would continue (Vallerand, 1997; Yoon and Rolland, 2012; Ryan and Deci, 2017). According to Ryan and Deci (2002). The sense of autonomy comes from an individual’s comprehensive self-awareness, controlled behavior stems from the causal relationship of external perceptions, and problem solving ability has proved to be an important factor in self-determination. A sense of relatedness can improve one’s ability to successfully respond to social situations, enhance the connection between different positive results, and increase participation and involvement in behavioral activities (Watanabe and Sturmey, 2003; Jang et al., 2016).

Self-determination theory assumes a set of three basic psychological needs—autonomy, competence, and relatedness. It is believed that meeting these needs will lead to greater intrinsic motivation and expectation of positive results, affecting whether individual behavior will continue and whether this behavior can be internalized into the psychological state of an individual’s self-discipline (Shir et al., 2019; Donaldson et al., 2021; Lu et al., 2021). For teaching activities of DDE, SDT can meet basic psychological needs and provide teachers with unique, meaningful backgrounds and opportunities related to new teaching methods, so that teachers can transform their work activities into more meaningful pursuits of their inherent growth and actively meet the need of their innate growth tendency (Ryan and Deci, 2017; Al-Jubari et al., 2019). Therefore, when participating in the teaching activities of digital entrepreneurship, teachers are given supports and stimulations to meet their needs for experience: they can organize their own goal setting and goal effort (autonomy), work on troubleshooting entrepreneurial activities (problem solving ability), and create meaningful relationships with students (relatedness). All of these needs can significantly affect the participation relationship in digital entrepreneurship teaching.

### Task-Technology Fit

Within the framework of personal or organizational work environment, the combination of work tasks and tool technology can be effectively reconciled with Task-Technology Fit (TTF), while TTF can encourage users to recognize the task context that affects their subsequent adoption behavior and improve their individual performance (Goodhue and Thompson, 1995; Zigurs and Khazanchi, 2008; Gay, 2016; Shafie et al., 2019). Instead of a direct impact, TTF works through the interaction between task and technology; different task characteristics will require different technological functions to assist. When the gap among the individual, technology, and task is small, TTF will increase (Goodhue and Thompson, 1995; Jang, 2016; Khan et al., 2018).

Digital entrepreneurship education is being incorporated into different research fields, including business, engineering, and science. Teachers are more important for interdisciplinary integration of knowledge and sciences, playing a vital role model for the overall effectiveness of DEE and helping students adapt to the new skills of changing environmental contexts (Nambisan, 2017; Steininger, 2019; Elia et al., 2020; Sahut et al., 2021), Otache (2019) pointed out that new forms of knowledge may be learned through face-to-face communication or other mechanisms that unobtrusively transfer knowledge. DEE further requires teachers to develop the ability to operate correctly with companies and to establish extensive network connections to make better use of market opportunities (Mitchelmore and Rowley, 2010; Bamiatzi et al., 2015; Geissinger et al., 2019). Teachers participating in DEE often specialize in business management, law, accounting, communication skills, and ICT tools. The development of DEE course content is therefore often influenced by dominant disciplines (such as marketing, finance, and accounting); as a result, DEE teachers tend to teach formulate operational plans and financial forecasts, relevant knowledge of start-ups, use of management tools, the ability to identify and analyze business opportunities, as well as activities and knowledge related to the forming of business literacy (Mitchelmore and Rowley, 2010; Morris et al., 2013; Geissinger et al., 2019; Garcez et al., 2021; Sahut et al., 2021). As the use of ICT increases, it is expected that more new technologies will subvert the existing business models (Giones and Brem, 2017; Nambisan, 2017; Ngoasong, 2018; von Briel et al., 2018; Garcez et al., 2021; Secundo et al., 2021). Therefore, DEE teaching should focus on how business literacy can match with the use ICT tool and create positive impact on the TTF between teaching tasks and technological tools.

As long as teachers can recognize the impact of ICT on the teaching and learning process of DEE, they will be more likely to start using ICT in their teaching and learning process (Wang et al., 2018; Rihtaršiè and Avsec, 2019; Elia et al., 2020; Saubern et al., 2020). Wang et al. (2018) and Saubern et al. (2020) suggested that teachers can effectively help their students develop their technical literacy only when teachers use ICT to support their teaching and learning methods, possess technical skills and abilities to teach, and have faith in teaching and their ability to learn professional knowledge. Reading and Doyle (2013) and Reyes et al. (2017) studied the factors related to the integration of ICT into teaching activities and cooperation, proving that these factors contribute to the driving force for teachers to develop their technical pedagogical content knowledge (TPACK).

### Hypothesis Development

Studies have considered SDT as the main pre-variables of teaching activities (perceptual autonomy, perceptual competence, and perceptual relatedness). Perceptual autonomy involves the mutual behavior happening when an actor promotes the intention and psychological needs of the receiver (Oosterbeek et al., 2010; Al-Jubari, 2019; Al-Jubari et al., 2019; Chung and Lee, 2020; Donaldson et al., 2021). When teachers have a sense of autonomy in their behavior, they will be more likely to organize their own learning over the process of DEE activities, set up and pursue goals of medium-to-high difficulty, and use all of their resources, talents, interests, and energies as the source of independent motivation for learners (Ryan and Deci, 2017; Baluku et al., 2018; Otache, 2019; Keyhani and Kim, 2020). Moreover, it is necessary for DEE teaching to include interdisciplinary literacy and technology and enhance learners’ problem solving ability as a result. This ability will enable teachers to take action on challenging tasks and have better work control to reduce their pressures from work. Self-motivation mechanisms and continuous activities can provide teachers with opportunities to solve entrepreneurial teaching tasks in their own way (Ismail et al., 2018; Ozgenel, 2018; Al-Jubari, 2019). Perceptual relatedness depends on the extent to which teaching behavior is correlated with behavioral activities. Perceptual relatedness can turn teachers into facilitators in the process of creating value with their students and innovating their teaching content and make teachers hope to become a member of the DEE teaching community and contribute to the social group they identify with (Baeten et al., 2013; Haivas et al., 2013; Al-Jubari et al., 2019). Fore et al. (2015) used experiential teaching to test teachers’ acceptance of new teaching methods, in which a sense of autonomy and relatedness allows teachers to perform better in teaching and have a longer-lasting motivational experience. In summary, the intrinsic value of these three basic needs is very important, because teachers will maintain positive results when their needs are satisfied. In terms of the internalized process of motivation, when teachers come to realize the values of what they do, identify with these values, and then find the results to be positive, DEE teaching activities will become more attractive to teachers, and they will decide to implement these activities accordingly. Based on the discussion above, the following hypotheses were proposed:

H1: Personal sense of autonomy (for teachers) has an impact on the positive attitude of DEE teaching;

H2: Personal problem solving ability (for teachers) has an impact on the positive attitude of DEE teaching; and

H3: Personal sense of relatedness (for teachers) has an impact on the positive attitude of DEE teaching.

When the spirit of entrepreneurship is boosted by business motivation to take risks, initiate and maintain profitability, and create goal-driven ventures, students will be given entrepreneurial tools and opportunities for implementation. In terms of business activities, Pittaway and Cope (2007) suggested that the development of business models, business plans, and entrepreneurial education can enhance learners’ understanding of a company’s operation, technology, finance, budget, and marketing capabilities and encourage them to transform their ideas of entrepreneurial activities into business propositions (Mitchelmore and Rowley, 2010; Fellnhofer, 2019; Kakouris and Liargovas, 2021). In digital entrepreneurship, it is necessary for entrepreneurial education to help learners develop literacy related to the virtualization of business process and business management, create businesses models that treat customers as value-creating, and use a huge user base to generate high network traffic. Learners should also know how ICT changes according to business models and process configurations in order to take advantage of market opportunities (Bechard and Gregoire, 2005; Shabbir et al., 2016; Steininger, 2019; Ratten and Jones, 2021; Sahut et al., 2021).

Digital literacy is generally defined as the integration of knowledge, skills, and attitudes related to the use of digital technology in daily life, which links together tool technology, media literacy, information skills, and computational thinking (Wang et al., 2018; Steininger, 2019; Saubern et al., 2020; Crosthwaite et al., 2021). Digital literacy can increase learners’ sensitivity of information availability and market knowledge, and teach them how to protect digital products and digital services against plagiarism and the challenge of new product liability. Moreover, digital literacy can use ICT to transform the scarcity, inimitability, and irreplaceability of digital resources into a competitive advantage (Nambisan, 2017; Ngoasong, 2018; Rihtaršiè and Avsec, 2019; Steininger, 2019; Vinogradova et al., 2019; Zaheer et al., 2019). Teachers can use ICT and new technical standards, select the best technical paradigm to reshape their courses, realize the specific teaching goals of DEE, integrate technology, teaching, and content knowledge, and promote the TTF of DEE teaching activities (Nambisan, 2017; Wang et al., 2018; Vorbach et al., 2019). Based on the discussion above, the following hypotheses were proposed:

H4: Personal business literacy (for teachers) has an impact on the TTF of DEE teaching, and

H5: Personal digital literacy (for teachers) has an impact on the TTF of DEE teaching.

In the teaching process, teachers tend to have a greater sense of autonomy, a better problem solving ability, and a clearer sense of relatedness, with enhanced positive attitudes toward digital entrepreneurship teaching (Ryan and Deci, 2017; Shir et al., 2019; Donaldson et al., 2021; Lu et al., 2021). The interdisciplinary nature and complex content of digital entrepreneurship can increase teaching content and the integration of technological tools into teaching activities. This suggests a stronger demand for supporting teachers’ personal psychological success, a significantly stronger sense of competence, and an expectation for positive results of course content design (Fellnhofer, 2019; Iwu et al., 2019; Vorbach et al., 2019; Lu et al., 2021). Therefore, with the enhancement of positive attitudes, teachers can continue to obtain more inner self-motivation. Based on this positive self-motivation, teachers can better plan on their teaching activities, prepare for different teaching situations, quantitatively evaluate the increased effect of teaching activities, and eventually increase their teaching intention.

H6: In DEE teaching, positive attitudes have an impact on teaching intention.

Discussions on the degree of coordination between tasks and technology are not limited to behavioral activities; they further explore the impact on performance. When the technology used can support task characteristics, the energy and costs spent on performing the tasks of digital entrepreneurial activities can be reduced. TTF has an impact on the performance of the behavior results, which can make a task progress more smoothly; this can reduce the energy and costs that the user spends on performing the task, making it easier to complete the task (Goodhue and Thompson, 1995; Gay, 2016; Zaheer et al., 2019; Crosthwaite et al., 2021; Ye, 2021). On the other hand, the multiple purposes of DEE teaching require teachers to use ICT tools to complete the tasks of their teaching activities. This shows that better TTF can result in better performance (e.g., Zigurs and Khazanchi, 2008; Jang, 2016; Khan et al., 2018; Shafie et al., 2019; Steininger, 2019). By extension, when teachers’ digital literacy can support them to make full use of ICT tools, match the business literacy of their personal task characteristics, and achieve the set performance goals of their teaching activity, their teaching activity will have a better TTF and consequently better improve their DEE teaching intention.

H5: The TTF of DEE teaching has an impact on teaching intention.

Digital technology has made it possible for entrepreneurs to develop and adjust their potential digital business ideas. It is now also possible for emerging digital technologies to support entrepreneurial learning experience, thereby providing DEE with better support (Otache, 2019; Elia et al., 2020). The participation of teachers and students, which is based on the learning activities and their interaction in the course activities, provides students with information about the available technologies for knowledge exchange and communication, supports them to familiarize themselves with digital tools and their functions, and promotes frequent communication between team members and lecturers. Teachers and students are thus encouraged to have knowledge exchange, make decisions based on their consensus, and create caring connections between learning communities and learning partners (Seikkula-Leino et al., 2010; Baeten et al., 2013; Haivas et al., 2013; Keyhani and Kim, 2020). As teachers and students interact in the entrepreneurial activities they participate in, teachers will change their roles, becoming supporters to students and working together with students in digital entrepreneurial activities (Bechard and Gregoire, 2005; Ismail et al., 2018; Iwu et al., 2019). Given access to students’ views on issues concerning digital entrepreneurship, teachers will become proactive collaborators with students able to integrate multiple perspectives to optimize their insights. This will have positive influence on teachers’ intention to teach digital entrepreneurship and help them implement DEE teaching activities more effectively.

H8: Interactive participation in DEE teaching has an impact on teaching intention.

The discourses of the related hypotheses were used to construct a theoretical model of this research (Figure 1).

**FIGURE 1:** Research framework.

## Data and Methods

### Research Design and Sample

Digital entrepreneurship education is implemented through Internet and digital technology platforms to manage and execute business activities with customers, intermediaries, and business partners. Virtual enterprises can be established by sales of digital products or services through the Internet and by Internet-driven business and business expansion (Shabbir et al., 2016; Steininger, 2019; Sahut et al., 2021). The sample population of this study was based on a selection of universities that have at least five departments or graduate programs related to business management and information technology and claim to have DEE activities on the University Course Resource Website of Taiwan^1^. As the selection criteria of participants required, teachers were invited only if they had taught courses on basic concepts of entrepreneurship, professional business, or comprehensive entrepreneurial management. The first phase used snowball sampling program to obtain a sample of 210 participants, who were sent a questionnaire on their intention to offer a DEE course. The questionnaire was sent to them either as a mail survey or an email form to fill in, and responders were asked to provide their email contact information and those of other potential participants. In the first phase, only 39 valid questionnaires were collected. The status of responses was not satisfactory, so the researcher contacted those who did not respond last time and 400 new potential participants in the second phase. Three weeks later, 87 valid questionnaires were collected. Among all the valid questionnaires, 66 were from male teachers and 60 were from female teachers. The youngest of the respondents was 28, the oldest one was 62, and the average age was 42.98 years. The standard deviation was 8.982 years. The basic information of the valid questionnaires is shown in Table 1. None of the participants were paid for their participation, and the questionnaire items were randomized together with items concerning individual performance. The data of each participant were processed anonymously, and the data of their responses are kept in a proper way that strictly abides by the anonymity requirements by Taiwan Academic Ethics for investigation and research.

**TABLE 1:** Profiles of participants (*N* = 126).

Demographics/Level	First	Second	Significant
**Gender**			
Male	22	44	Chi-square = 0.368
Female	17	43	*p*-value = 0.544
**Digital entrepreneurship education experiences (years)**			
One	13	20	Chi-square = 1.676
Two	15	42	*p*-value = 0.433
Three	11	25	
**Course count**			
One	15	41	Chi-square = 3.201
Two	9	17	*p-*value = 0.669
Three	4	14	
Four	4	4	
Five	6	9	
Missing value	1	2	
**Age**			
Mean	44.23	42.41	*t*-value = 1.050
*SD*	7.949	9.938	*p*-value = 0.296

### Variables and Measures

The impact of ICT tools and digital technologies on business innovation and entrepreneurship is multifaceted. In digital entrepreneurial activities, they can be the promoters of entrepreneurial operations; they can even dominate the overall business model. This study drew from past literature of entrepreneurial education and DEE, selected literature related to business and digital literacy, SDT, TTF, and developed relevant measurement items. All the items were measured on a 7-point Likert Scale, ranging from “strongly agree” (7 points) to “strongly disagree” (1 point) and from “strongly willing to” (7 points) to “strongly unwilling to” (1 point). The operational definitions are listed in Table 2.

**TABLE 2:** Operational definition of variables.

Dimension/Variable	Operation definition	Literature
Autonomy	A teacher’s self-determination to engage in DEE teaching activities, along with his/her initiative and effort in the process of the activities.	Ryan and Deci, 2017; Al-Jubari et al., 2019; Otache, 2019; Keyhani and Kim, 2020
Problem solving ability	A teacher’s ability to manage the teaching activities of DEE, control the teaching work, motivate himself/herself, adequately and effectively perform the teaching activities, and effectively produce anticipated results and prevent adverse consequences.	Ryan and Deci, 2017; Ismail et al., 2018; Ozgenel, 2018; Al-Jubari et al., 2019
Relatedness	The association between a participant’s behavioral activities and DEE teaching, which makes him/her become a member of the digital entrepreneurship teaching community and a contributor to the social group he/she identifies with.	Baeten et al., 2013; Ryan and Deci, 2017; Al-Jubari et al., 2019
Positive attitude emotions	A participant’s feeling of preference and positive emotions for DEE teaching activities, with behavioral results expected to bring pleasant feelings.	Jang et al., 2016; Ryan and Deci, 2017; Al-Jubari et al., 2019; Shir et al., 2019; Chung and Lee, 2020; Donaldson et al., 2021; Lu et al., 2021
Digital literacy	The ability to use knowledge and skills required master the technological tools required by DEE teaching activities, mainly for teachers to understand the characteristics of technological tools as well as to select, find, and evaluate tools and technical resources more effectively.	Guthrie, 2014; Giones and Brem, 2017; Ngoasong, 2018; Rippa and Secundo, 2019; Steininger, 2019; Vinogradova et al., 2019; Elia et al., 2020; Saubern et al., 2020; Crosthwaite et al., 2021
Business literacy	The ability to master business knowledge and skills required by DEE teaching activities, mainly for teachers to effectively select, find and evaluate market opportunities, corporate governance, production and service activities, financial activities, etc.	Mitchelmore and Rowley, 2010; Shabbir et al., 2016; Ozgenel, 2018; Geissinger et al., 2019; Garcez et al., 2021; Sahut et al., 2021
Task-technology fit	The accuracy, ease of acceptability, flexibility of the user interface, assistance, credibility of the technology tools provided by the technology tools to complete the DEE teaching activities after the collocation of business and digital literacy.	Gay, 2016; Jang, 2016; Reyes et al., 2017; Khan et al., 2018; Shafie et al., 2019; Steininger, 2019
Interactive participation	A teachers’ willingness to share information, work on interpersonal communication, invest his/her personal resources, encourage students, and continue to interact with his/her peers and students in DEE teaching activities.	Nambisan, 2017; Ismail et al., 2018; Jones et al., 2018; Keyhani and Kim, 2020
Teaching intention	A teacher’s subjective determination to start a DDE course, based on his/her personal belief that the course outcome and learning results brought by DEE courses will exceed expected results or create a high degree of satisfaction.	Guthrie, 2014; Jang et al., 2016; Ismail et al., 2018; Al-Jubari et al., 2019; Otache, 2019; Keyhani and Kim, 2020
Demographics	Demographic variables are mainly individual demographic variables	
Age	The age of the teacher interviewed	
Sex	The sex the interviewed teacher	
DEE teaching experience	A teacher’s experience in DEE and the number of DEE courses he/she has taught within a year.	

### Analytical Procedures

In order to avoid potential problems related to common method variance (CMV), the anonymity requirement for the participants was declared in the answering instructions of the questionnaire, the participants were clearly told that there were no correct or wrong answers to any question, and the questionnaire items were processed in a random fashion. With these three steps, the research tried to reduce the respondents’ fear of participating in the questionnaire and make it less likely that the respondents might answer the questionnaire in a socially expected way. In order to understand whether the collected samples were representative and without any non-response bias, the study adopted the chi-square or *t*-test between early respondents and late respondents. Early respondents were defined as participants in the first phase of questionnaire collection. Participants in the second phase included late respondents and participants who did not complete the survey. Then four indicators—the demographical factors of sex and age, DEE teaching experience, and the number of DEE courses offered last year—were compared between the first-phase respondents and the second-phase respondents. No significant difference was found (*p*-value > 0.05). The verification results are shown in Table 1.

## Results

### Measurement Model

This study adopts SmartPLS3.0, developed by Ringle et al. (2015), as its data analysis software system to analyze the measurement model and structure model. The bootstrapping sample was set to 3,000 times. Based on the recommendations of Hair et al. (2011), this study selected five most commonly used indicators to evaluate the measurement mode of reflective indicators. Each indicator is described as follows:

Individual item reliability: This indicator evaluated the factor loading of the measured variables on the potential construct. The factor loading coefficient of the tested sample was between 0.741 and 0.948, and the load of each measurement variable was greater than 0.6 and has statistical significance (Hair et al., 2011).

Composite reliability (CR) of potential variables: The CR value of potential variables is the composition of the reliabilities of all the measured variables. Its index meaning is similar to Cronbach’s Alpha, which is used to express the internal consistency of the construct index. The CR value of the measured sample ranged from 0.876 to 0.946. The internal consistency of this research model was good, and it also met the recommended value of Chin (1998)—to be greater than 0.7. When measured by the customary Cronbach’s Alpha coefficient, the construct of Cronbach’s Alpha in this study was between 0.814 and 0.928, also higher than the general requirement for Cronbach’s Alpha—to be greater than 0.7 (Nunnally and Berstein, 1994).

For the rho_A reliability index, this study did not use factor loading to calculate the consistency of the construct. According to the Dijkstra and Henseler (2015) literature, it used the least squares method to reproduce the correlation matrix of the measurement items; the better the result was, the higher the coefficient value would be. The rho_A of this study ranged from 0.831 to 0.929, which showed that construct internal consistency of this study was good.

Average variance extracted (AVE) of potential variables: A higher AVE value means both discriminative validity and convergence validity of the potential variables are better. In this study, the AVE value of each potential variable in the tested sample ranged from 0.639 to 0.883, higher than the standard value (0.5) recommended by Fornell and Larcker (1981). Relevant information is shown in Table 3.

**TABLE 3:** Validity and reliability of research model.

	Mean	*SD*	Cronbach’s alpha	rho_A	Composite reliability (CR)	Average variance extracted (AVE)
Autonomy	4.903	1.223	0.901	0.903	0.926	0.716
Relatedness	5.537	0.811	0.866	0.938	0.904	0.703
Problem solving ability	5.421	1.099	0.819	0.825	0.873	0.579
Digital literacy	5.526	0.957	0.875	0.885	0.910	0.669
Business literacy	5.158	1.032	0.853	0.879	0.900	0.693
Positive attitude emotions	4.966	1.071	0.867	0.868	0.905	0.656
Interactive participation	5.176	1.003	0.816	0.867	0.867	0.568
Task-Technology fit	5.372	1.110	0.877	0.884	0.916	0.732
Teaching intention	5.472	0.931	0.905	0.908	0.930	0.725

The measurement model needs to be tested for discriminant validity (Henseler et al., 2015). According to Fornell and Larcker (1981), the root mean square of each construct of AVE is greater than the correlation coefficient between construct pairs. As shown in Table 4, the root mean square of all dimensions of AVE was greater than the correlation coefficient between different dimensions, so this study had sufficient discriminative validity.

**TABLE 4:** Discriminative validity (Fornell and Larcker criteria) of research model.

	Autonomy	Relatedness	Problem solving ability	Digital literacy	Business literacy	Positive attitude emotions	Interactive participation	Task-Technology fit	Teaching intention
Autonomy	0.846								
Relatedness	0.446	0.839							
Problem solving ability	0.510	0.285	0.761						
Digital literacy	0.796	0.602	0.528	0.818					
Business literacy	0.492	0.628	0.394	0.658	0.832				
Positive attitude emotions	0.664	0.464	0.491	0.626	0.578	0.810			
Interactive participation	0.712	0.599	0.448	0.644	0.574	0.650	0.754		
Task-Technology fit	0.660	0.584	0.539	0.719	0.649	0.662	0.644	0.856	
Teaching intention	0.551	0.498	0.499	0.504	0.359	0.530	0.560	0.553	0.852

*Diagonal element is square root of AVE and should be larger than the off-diagonal correlation coefficient.*

### Structural Model

The structural model path analysis coefficients for SDT exogenous variables into teachers’ positive attitude emotions were as follows: Autonomy - > Positive attitude emotions (0.479); Problem solving competence - > Positive attitude emotions (0.190); Relatedness - > Positive attitude emotions (0.197). All of them reached the significance level α = 0.01 and supported H1–H3. Then, the path coefficients for individual literacy to teachers’ task-technology fit—Business literacy - > Task-technology fit (0.310), Digital literacy - > Task-technology fit (0.515)—reached the significance level α = 0.01 and supported H4–H5. Finally, the path coefficients of antecedent variables for teachers’ teaching intention were as follows: Positive attitude emotions - > Teaching intention (0.180); Task-technology fit - > Teaching intention (0.255); Interactive participation - > Teaching intention (0.279). These three paths reached the significance level α = 0.05 and supported H6–H8. The model explained of the variance in the endogenous variables: Positive attitude emotions for 50.3%, Task-technology fit for 57.1%, and Teaching intention for 39.2% (see Figure 2 and Table 5).

**FIGURE 2:** Results of the structural model testing. Value on path, standardized coefficients (β); *R*^2^, coefficient of determination. *p < 0.05; **p < 0.01.

**TABLE 5:** Estimation results for hypotheses.

	Path coefficient	*T*-values	*P*-values	Hypotheses
Autonomy - > Positive attitude emotions	0.479**	5.940	0.000	H1 support
Problem solving ability - > Positive attitude emotions	0.191**	2.699	0.007	H2 support
Relatedness - > Positive attitude emotions	0.197**	2.971	0.003	H3 support
Business literacy - > Task-Technology fit	0.310**	3.439	0.001	H4 support
Digital literacy - > Task-Technology fit	0.515**	6.541	0.000	H5 support
Positive attitude emotions - > Teaching intention	0.180*	2.034	0.042	H6 support
Task-Technology fit - > Teaching intention	0.255*	2.015	0.044	H7 support
Interactive participation - > Teaching intention	0.279*	2.334	0.020	H8 support

*p < 0.05, **p < 0.01.

## Discussion

### Theoretical and Practical Implications

It is most appropriate for universities to include DEE. Teachers may be voluntary or may be driven by certain purposes when they become engaged in digital entrepreneurship teaching activities. It is very important to have a better understanding of the motivation process of teachers’ intention to engage in digital entrepreneurship. This study integrated SDT and TTF, offering a supplementary explanation to the motivation process of entrepreneurship teaching activities—teaching intention, with *r* square = 39.2%. As an investigation on how digital entrepreneurship and technology can be integrated into teaching, this study shows results that are consistent with those of previous research in the context of teaching activities integrated with technology (Holland and Piper, 2014; Jang, 2016; Khan et al., 2018; Rippa and Secundo, 2019; Shafie et al., 2019; Chung and Lee, 2020; Secundo et al., 2021). This result provides a brand-new path for research on digital entrepreneurship and teaching activities that integrate professional literacy into the use of scientific and technological tools.

From the perspective of the SDT model, when teachers’ sense of autonomy, problem solving ability, and their sense of relatedness are enhanced, teachers will be positively motivated by some psychological mechanism to enhance their exposure to DEE and their acceptance of DEE-related courses. This shows that autonomy, relatedness, and problem solving ability can strengthen teachers’ personal positive emotions, encourage them to work on innovation, entrepreneurship and appropriate adjustments to the content of teaching materials, and eventually enhance their teaching intention (Al-Jubari, 2019; Al-Jubari et al., 2019; Chung and Lee, 2020; Donaldson et al., 2021; Lu et al., 2021). In the theoretical model, autonomy is still the strongest factor, which, significantly supported by statistic data, shows that the stronger teachers’ sense of autonomy grows, the stronger and clearer their positive attitude toward DEE teaching will become. This research result is consistent with those of previous SDT research on teaching activities (Baluku et al., 2018; Otache, 2019; Shir et al., 2019; Keyhani and Kim, 2020). As teachers have more positive emotions in their courses, their willingness to teach digital entrepreneurship courses will also increase. This is shown by their continuous investment in entrepreneurship courses and their willingness to continue the courses (such as Iwu et al., 2019; Shir et al., 2019; Donaldson et al., 2021).

In the course of teaching, these teachers need to have digital literacy in new ICT tools and business literacy for entrepreneurship. Mission-oriented business literacy and digital literacy of technology tools are supported by empirical data in this study. The business literacy and digital literacy of teachers are statistically significant for TTF. This result is consistent with those of previous research on digital entrepreneurship research (e.g., Jang, 2016; Nambisan, 2017; Khan et al., 2018; von Briel et al., 2018; Vorbach et al., 2019; Elia et al., 2020). However, the present study was most affected by the teachers’ digital literacy in TTF (Guthrie, 2014; Nambisan, 2017; Vinogradova et al., 2019; Vorbach et al., 2019; Secundo et al., 2021). Mission-oriented business literacy (Bechard and Gregoire, 2005; Morris et al., 2013; Fellnhofer, 2019) has a low effect on TTF promotion. Technological tools can support the task activities of digital entrepreneurship teaching, improve learners’ pursuit of the benefit that digital entrepreneurship can be a profession, and stimulate learners’ awareness and pursuit of digital entrepreneurship. Teachers’ attentiveness can help reduce the energy and costs of performing digital entrepreneurial activities, allowing teachers to improve their teaching intention. This result is consistent with those of previous research on TTF (Holland and Piper, 2014; Gay, 2016; Reyes et al., 2017; Shafie et al., 2019; Crosthwaite et al., 2021; Ye, 2021). This study suggests that teachers should effectively improve students’ core skills rather than focus on professional business knowledge. This will have a practical impact on learners. Teachers need to modify their teaching techniques and curriculum content and improve personal teaching performance to optimize students’ acquisition of entrepreneurial knowledge.

The interaction between the instructor and the learners in the classroom learning process is of considerable significance. Teachers need to participate frequently in DEE program online, constantly give students advice and support students through online communication. Online communication can create stronger motivation for team members, improve their familiarity with each other, build their confidence in each other, and make them understand each other’s behavior, attitude, and professional knowledge, thereby encouraging them to exchange information and experiences (Seikkula-Leino et al., 2010; Haivas et al., 2013; Ismail et al., 2018; Iwu et al., 2019; Keyhani and Kim, 2020). The interaction between a teacher and his/her students is consistent with the development of learning activities, and the participation and interaction between the teacher and learners (sharing, discussing, reflecting, etc.) is helpful for learning effectiveness; it is also an intangible form of encouragement for teachers. This is consistent with results of previous research (Reading and Doyle, 2013; Ismail et al., 2018; Otache, 2019; Donaldson et al., 2021). Through the interactive participation of learners, teachers’ teaching intention can be strengthened, teaching goals can be achieved, and fruitful research results can be found. In the process of DEE teaching, teachers and students tend to learn together by doing and grow together by interacting with each other. This can increase the importance of DEE for teachers and strengthen their intention to teach DEE courses. The more interest teachers show in their teaching and the more they encourage students to participate in activities related to digital entrepreneurship, the more students will accept entrepreneurship.

When managers of educational institutions and government departments responsible for higher education seriously consider introducing DEE as a subject into university curriculum, teachers and students in universities and colleges related to entrepreneurship should begin interactive learning courses with experiments, experiential learning, teamwork cooperation, and constant interaction between teachers and students, in order to achieve the educational goals of DEE (Vorbach et al., 2019; Zaheer et al., 2019; Elia et al., 2020; Ratten and Jones, 2021). When teachers personally have more positive feelings for the digital entrepreneurship courses, their intention to start DEE courses will increase, their TTF will become better, and their connection with entrepreneurial network will be stronger. This will promptly lead to their continuous investment in entrepreneurship courses and their intention to continue the DEE courses. This research result is consistent with those of previous research on DEE teaching activities (e.g., Guthrie, 2014; Ismail et al., 2018; Al-Jubari et al., 2019; Keyhani and Kim, 2020). More important for digital entrepreneurship activities to fully optimize the impact of entrepreneurial initiative and economic development, diversify experiential teaching, integrate the environment of intensive knowledge fields and thinking structure, stimulate personal creative thinking skills. In the DEE courses, encouraging teachers’ enthusiastic participation in the teaching activities of digital entrepreneurship, designing business academic courses and ICT course content, and introducing technological tools to stimulate more opportunities for digital entrepreneurship.

### Limitations and Future Research

Future research on DEE should mainly focus on a broader interdisciplinary perspective brought by ICT tools, which can make digital entrepreneurship activities more rapid and complex. DEE should help learners develop their problem solving ability for digital business activities required by new market conditions.

#### First Research Limitation

The rapid change of ICT tools and technologies can overturn the technical utilities of teachers in certain fields of educational activities. For example, technologies that were described as emerging or less common 5 years ago may have been widespread today and have become effective. In pursuit of effective teaching, teachers may find that their competences tend to be easily outdated. In order to overcome this risk of rapid obsolescence for research results in future research, the focus should be on the development of capabilities and beliefs on the basis of the digital literacy in these technological tools, rather than simply on certain skills specifically used for current or emerging technologies.

#### Second Research Limitation

Concerning the investigation on teachers’ actual business literacy and digital literacy, this study mainly drew from teachers’ reports on their own competences, skills, and knowledge. Therefore, there is a risk of distortion of or deviation from the actual situations; that is, teachers might overestimate or underestimate their own levels of business literacy and digital literacy. In order to assess the validity and reliability of teachers’ descriptions of their own literacy levels, this study suggests that quantitative research should be conducted from different perspectives (triangulation) at the same time. For example, research should focus on teachers’ views of the use of technology in teaching and the extent to which teachers play a role model in this regard, while eliminating the interference effects brought by the learning environment and facilities required by ICT tools.

#### Third Research Limitation

The sample population of teachers interviewed in this study was limited by its setting that teachers were invited only if they had taught related courses in a selection of universities that claim to have DEE activities on the University Course Resource Website of Taiwan (see footnote 1). Moreover, the survey was conducted by a valid sampling of 126 teachers and is therefore not a survey study with a large number of samples. It is advisable that researchers, upon making theoretical generalization inferences, should also pay attention to the degree of generalization caused by the small number of samples, in addition to considering whether similar research is applicable to other regions or countries.

## Conclusion

Digital entrepreneurship education can educate students on entrepreneurship knowledge, make students familiar with ICT tools and the use of new technologies, increase professional digital entrepreneurship courses, and help students create online employment opportunities. For DEE teachers, it is a novel and challenging teaching activity to adapt to an interactive student-centered pedagogy that focuses on the practice of entrepreneurship. Based on the behavior patterns of teachers in offering DEE courses, this study proposes an effective theoretical framework to understand college teachers’ intentions to offer DEE courses. According to Self-determination theory, positive psychological incentives can encourage teachers to learn more about DEE and further enhance their willingness to offer DEE courses. The matching-up of teachers’ digital competence and business literacy can speed up the task of completing DDE teaching activities. Given the mutual participation and support of their community, individual teachers will be greatly inspired to enthusiastically participate in DEE courses. The teaching activities can be novel and challenging, with DEE’s integration of ICT tool technology and entrepreneurial activities. It is indeed a new thread for research on teachers’ behavior of offering DEE courses to understand the psychological processes of teachers being motivated by DEE courses and the digital competence and business literacy they should acquire and develop in order to complete the required teaching tasks of DEE.

## Data Availability Statement

The original contributions presented in the study are included in the article/supplementary material, further inquiries can be directed to the corresponding author/s.

## Ethics Statement

Ethical review and approval was not required for the study on human participants in accordance with the local legislation and institutional requirements. Written informed consent from the patients/participants was not required to participate in this study in accordance with the national legislation and the institutional requirements.

## Author Contributions

T-KY: research ideas, concept and design, obtaining funding, statistical analysis, interpretation of data, and study supervision. C-MC: data curation, concept and design, statistical analysis, interpretation of data, and writing up. YW: data curation and interpretation of data. All authors: wrote the manuscript together and approved the final manuscript.

## Conflict of Interest

The authors declare that the research was conducted in the absence of any commercial or financial relationships that could be construed as a potential conflict of interest.

## Publisher’s Note

All claims expressed in this article are solely those of the authors and do not necessarily represent those of their affiliated organizations, or those of the publisher, the editors and the reviewers. Any product that may be evaluated in this article, or claim that may be made by its manufacturer, is not guaranteed or endorsed by the publisher.

## Footnotes

1
https://ucourse-tvc.yuntech.edu.tw/WebU/index.aspx
